# Study on the Reform and Development of Modern Physical Education Teaching Based on 5G Internet Communication Technology

This article has been retracted.

**DOI:** 10.1155/2022/5604141

**Published:** 2022-05-16

**Authors:** Shaohui Du, Ning Han, Feng Yi

**Affiliations:** ^1^Physical Education Department, Jiangsu University of Technology, Changzhou 213001, Jiangsu, China; ^2^School of Sports and Health Engineering, Hebei University of Engineering, Handan 056038, Hebei, China

## Abstract

Physical education (PE) is, in general, one of the most important skills developed for human healthiness. Many barriers exist in society to improve the performance in Chinese physical activities. Furthermore, the incorporation of 5G communication network technology is becoming a trend in the increase of physical activity in China on a daily basis. Physical exercise may assist Chinese people to enhance their mental abilities, self-concept, and goal orientation and avoid mental illnesses such as sadness and anxiety. Physical exercise without education is like having a body but no soul. There is no doubt about the value of physical education and other types of exercise in the educational system. In this paper, we propose refined physical education teaching based on 5G network technology to obtain everlasting data without termination. First, we preprocess the sports dataset using a stacked denoising autoencoder (SDAE), and a Gaussian Mixture Model (GMM) is utilized for the feature extraction process. A random forest approach (RFA) is then used in the selection of the features. Furthermore, we adopted a CNN-based upgraded classifier for classification and efficient data allocation (EDA) algorithm for storing data generated by the 5G network. Experimental results reveal that our proposed method outperforms the baseline methods by a huge margin.

## 1. Introduction

Higher education reform has grown more in-depth, with the growth of education in universities and the deepening of changes taking place in this contemporary period. Since physical activity is an essential component of the educational process, the impact of physical activity on students' future health and educational development is closely tied to the future growth of the nation's health and education. There are various concerns with students' primary fitness education, according to the findings of this research, including the use of a conventional teaching strategy, the lack of a distant teaching technique, and the inability to conduct thorough technical evaluations. The demand for physical education material among college students is always growing in tandem with the overall expansion of society [1].

The primary goal of physical education instruction is to develop students' abilities in the areas of health and exercise. As a consequence, correct exercise routines and methods are essential components of the curriculum. The specialists have found a weakness in the traditional method of teaching physical education, who have discovered that the individual's emotional and physical traits are commonly disregarded [2]. A great deal of global research has been done on networked physical education, especially in the areas of digital learning and gamification. Its primary goal is to improve educational quality via the use of existing network devices and network connection modes, which are already in place. A significant effect has been achieved during the COVID-19 era by interconnected primary fitness education, which has the ability to enhance and increase instructional efficiency in a very short amount of time. Physical activities that are part of a network, on the other hand, are more generally acknowledged than traditional physical education. Therefore, it is critical to develop digital physical education by allowing interconnected physical education to have adaptive features, increase latency, and experience quality [3] and establish digital physical education infrastructure.

The approach of physical education is influenced by a variety of aspects. The AI and machine vision can be implemented to support and construct physical education tasks, which increase the effectiveness of physical education and give a comprehensive teaching assessment method for the physical education system [4]. Implementing computer-assisted instruction (CAI) in the area of physical training is a critical step in moving away from the usual framework towards the research and information, and it is one of the most difficult in the field. Artificial Information technology plays a vital role in computer-assisted training, and the integration of CAI and AI will enhance the teaching methods in such a manner that people can easily distinguish the module's teaching material, teaching topic, and teaching approach. The method and composition of physical education are based on information input from the student's learning theory, can be easily differentiated in that way, achieve the AI system contents and logic, and typically influence physical teaching material and educational methods that lead to individual distinctions [5].

The rest of this article is structured as follows.  Section 2 offers the literary works associated with this paper.  Section 3 explains the proposed model.  Section 4 provides the performance analysis of the suggested method. And, finally, Section 5 concludes the overall idea of the paper.

## 2. Related Works

District standards for smartphones, such as lower information rate gadgets, power consumption, and the gadget of things, were proposed by Lei et al. [6] and are analogous to Long-Term Evolution guidelines (LTE). Various Internet of Things standards under development could help with this problem. Its function is a vital component of the fifth-generation cellular network's future networking capabilities, which will replace the earlier smartphone's customary restriction. Physical health, according to studies, is helpful to both students and the greater society. The first step in achieving this aim is to improve one's overall physical condition. Physical education may help children improve social skills such as flexibility, response time, speed, collaboration, balance, and basic physiological movement, among other things. Zhan [7] studied IoT and healthcare and physical activity solutions. Existing research should be categorized and made available in the fifth-generation medical framework. In certain cases, healthcare and physical activity are also required for the successful integration of the fifth generation. Finally, numerous critical themes will be explored, including the limitations of researching the Internet of Things, fifth-generation healthcare, and physical exercise.

Cheng [8] proposed that data from a device's decision-making process be matched to off-the-shelf standards to establish an assessment and collective physical education process. The use of genetic algorithms is to augment reality for educational and training purposes. Virtual Reality (VR) development in this field is based on practical instruction and preparation. VR's original features and distinguishing characteristics might be extensively employed in practical training, with preparation playing a critical part. The embedded system is an important component of today's electrical components. Embedded equipment often operates as a single program and communicates with other network devices through a network connection. As a consequence of the equipment requirements, users get some expertise in the digital world. It is a big step forward in the evolution of VR.

Li and Tsai [9] investigate the digital network classroom approach as a university physical fitness learning model. The University of Physical Fitness Teaching Method in the digital classroom network may greatly guide and boost student learning interests and motivation. As a result of digital classroom networks, more instructors are recognized and engaged in physical exercise. The creation of a university physical activity evaluation procedure should include fifth-generation digital network generation elements. The exploration-based college physical education assessment technique is more objective than the current approach. Therefore, it is conceivable to analyze college PE using a 5G digital network. Zhu [10] investigated changes in people's daily exercise routines and body composition as a result of previous and initial educational reforms, and we presented a combination of educational reforms and an experiment with digital integration using fifth-generation cloud computing communication technology. The following processes were employed: a study of the literature, questions, a teaching experiment, measurement, and quantitative statistics. The results of the digital fusion and combined education reform experiment with fifth-generation cloud computing communication technology show that education transformation can increase the number of university students who participate in sports while also influencing changes in their body composition. As a consequence, in the reform of physical education programs, a digital teaching technique based on fifth-generation cloud computing communication technology is inescapable. It may assist students in not only developing physical fitness, but also in improving their health to some extent. As a consequence, it backs China's great health policy. Chen and Liang [11] advocated transforming the martial arts education system by using cutting-edge 5th generation technology.

Technology has improved training and provided essential PE gaming skills. Sun and Gao [12] developed a way to construct a new digital teaching approach for physical education. For starters, edge computing for PE may improve management system efficiency. Second, a backpropagation neural network with particle swarm optimization is used to evaluate data from college physical education management approaches. Finally, tests reveal that the approaches can easily edit, remove, search, and enter data, allowing the university sports department to manage physical education resources digitally. Du and Nan [13] proposed an ANN system based on accelerometer readings. A thorough analysis of technologies with potential commercial products based on the FPGA tool compares this research with the current development progress. Technological developments have improved education and provided PE gaming abilities. Motion tracking devices may help enhance athletic teaching skills by predicting people's location availability. Xu et al. [3] investigated 6CNRD, a novel framework connected to IPv6 Content Networking, to help create PE (6CN). 6CNRD has two stages: content delivery (identity forwarding) and content request (segment routing). We compare 6CNRD to two cutting-edge approaches across a planned physical education topology, and 6CNRD has fewer delivery delays and routing. It also reveals that 6CNRD is useful outside of physical education. Wang et al. [14] developed a cloud-based and wristband-based technique for group-centric physical education assistance. These operations are divided into three phases based on event streams: Internet of Things node networking and setup before class, real-time health monitoring and emergency scenario detection during class, and student progress and standard course evaluation after class. A method is also designed to educate and compare our proposed approaches to other methods.

Chao and Gang [15] use cloud computing and big data questionnaire survey, data analysis, experimental research methods, and data statistics. Experiments have shown that merging Big Data and Cloud Computing may overcome conventional teaching problems, allowing for efficient and rapid progress. According to Kaiyan and Qin [16], the national fitness program has increased the number of people engaged in physical exercise. A lack of public sports facilities hampers sports development. Also, this study stresses a network platform of all university sports venues resources that may support national fitness. The findings show the network platform's durability, concurrency, and practicality in the big data age. People's activity patterns have changed in the era of big data, as shown by Yu et al. The advent of the big data age will trigger considerable changes in university education. Big data may be used to enrich coaching approaches, subjects, and methods to inspire students to study sports more deeply. As a consequence, this article will concentrate on reforming university PE in the age of big data. Dong [17] investigated a big data embedded system to improve the efficiency of teaching physical skills and fulfill the demand for highly trained athletes. This research examines the significance of big data and embedded system approach to assess the college physical activity coaching information system about the big data mobile terminal. Sun [18] focused on the adjustments of university sports based on AI and IOT technologies to university Physical education management. The phrase “smart sports” refers to a notion that addresses both human and sporting needs. I think it is a great concept for China's future sports development and becoming a sports power.

## 3. Proposed Work

China released a study on the use of 5G technology in physical education, signaling the start of the fifth generation-enabled physical education era [19]. The goal of 5G-enabled physical education is to promote “physical education” and how to properly assist teens' physical activity habits development. This section describes how the recommended approach works.  Figure 1 depicts a schematic illustration of the proposed technique.

### 3.1. Dataset

The PAMAP2 dataset was compiled from the data of ten individuals (seven men and three women) who participated in 18 different physical activities. The subjects ranged in age from 27 to 31 years, with a body mass index ranging from 25.11 to 2.62 kg. They were all female. All of the participants, with the exception of one who was sinistral, were right-handed. Three inertial measurement units (IMUs) and a heart rate monitor were employed as sensor units to gather data. Three Inertial Measurement Units (IMUs) were implanted on the subject's body at three different locations: the hand, the chest, and the ankle. Each IMU is equipped with a three-axis gyroscope, a three-axis magnetometer, and two three-axis accelerometers, all of which operate at the same sampling frequency [20].

### 3.2. Data Preprocessing Using Stacked Denoising Autoencoder

The input and hidden layers of numerous denoising autoencoders are stacked in the stacked denoising autoencoder (DAE). DAE consists of three layers: hidden layer, input, and an output layer that uses encoders and decoders to obtain the output. To learn hidden features, the encoder can encode input data. The decoder can then decode the encoder's output and reorganize the data. Its purpose is to keep input and output as stable as possible while minimizing their loss. In addition, a denoising factor is utilized to corrupt input to prevent the problem of output being a straight copy of raw input. The stacking denoising autoencoder training method is subdivided into two parts:

- pretraining
- fine-tuning.

#### 3.2.1. Pretraining

In this step, the stacked denoising autoencoder employs layer-wise learning to enhance the specification of the denoising algorithm. The training of each denoising autoencoder in a stacked denoising autoencoder is done independently of the others. Furthermore, each DAE output will serve as an input to a future denoising autoencoder until the complete network has been trained. In order to train a denoising autoencoder, the two phases of encoding and decoding must be completed. The sigmoid function, which is used to compares data, will be used to transfer our training data to a hidden layer in the encoding process, and the sigmoid function will be used to decode the data from the hidden layer.

Formally, let *c*_*i*_ denote the input data, which have been previously classified and segmented and *c*_*i*_  is a 1 *∗* *M* vector. In this paper, the *M* equals 3071. The whole dataset is denoted as follows:

(1) $$\begin{array}{c} P_{a}=\left\{c_{0},c_{1},\ldots ,c_{a}\right\}. \end{array}$$

Firstly, each *c*_*i*_′ is corrupted by a denoising factor *a*, which obtains *c*_*i*_′. The possibility of every node lost in the layer is *a*. The encoding section *c*_*i*_′ is mapped to the hidden layer by a sigmoid function *s*, namely,

(2) $$\begin{array}{c} \;d=h\left(V_{1}c_{i}^{\prime }+b_{1}\right), \end{array}$$

where  *V*_1_ and  *b*_1_  denote the bias and weight matrix. Afterward, the *x* is mapped to the output layer by a sigmoid function *f*, namely,

(3) $$\begin{array}{c} \;z=g\left(V_{2}x+b_{2}\right), \end{array}$$

where  *V*_2_ and  *b*_2_ denote the bias and weight matrix, respectively. The inaccuracy between the generated data and the raw data is then estimated. The cross-entropy loss function is used, which is expressed as

(4) $$\begin{array}{c} \left(c_{i},z\right)=-\overset{a}{\underset{i=0}{\sum }}\left(c_{i}\log\right.\left(z\right)+\left(1-c_{i}\log\left(1-z\right)\right). \end{array}$$

Finally, gradient descent is used to update the parameters of each layer. The pretraining procedure is then completed.

#### 3.2.2. Fine-Tuning

In this phase, a softmax layer is added to the beginning of the network, which is then used to determine the activity occurring. Following that, the complete network would be trained in a supervised manner using labeled data, similar to how a multilayer perceptron would be trained (MLP). It is important to note that the pretraining process criteria are related to the fine-tuning process and that this is true. Following that, backpropagation and gradient descent is used to fine-tune the parameters of each layer in the network. During the training phase, the whole dataset is proportionately partitioned into three sets, training, validation, and test sets, respectively.

### 3.3. Feature Extraction Using Gaussian Mixture Model

Because a Gaussian Mixture Model can deal with a multimodal background, it is often used to detect physical motions in data. It calculates the value of each pixel by taking the mean and variance of all the sample pixels and averaging them together. With each frame, a new Gaussian Mixture Model pixel is produced and updated, resulting in a total of 256 pixels. Some of the Gaussian components match the current value at each new frame, and the running average updates the mean and variance for those components.

#### 3.3.1. Gaussian Mixture Model Updating

GMM contains three parameters that, one by one, update the pixels and frames. The parameters are the mean, covariance, and mixing parameters.

#### 3.3.2. Mathematical Proof of the Gaussian Mixture Model

This section describes the mathematical proof of the GMM. The three major parameters of a GMM are covariance, mean, and mixing parameter. We show how to change these three settings correctly in these instances.

#### 3.3.3. Learning Gaussian Mixture Models

The GMM *G*(*v*)=(*c*_*i*_(*v*))_*i*=1^*m*^_ is a finite collection of m-sized clusters, each of which is given at the tth instant.

(5) $$\begin{array}{c} \;A_{i}\left(\text{v}\right)=\left({µ}_{i}\left(v\right),\delta_{i}\left(v\right),\pi \left(v\right)\right), \end{array}$$

where *µ*_*i*_(*v*), *δ*_*i*_(*v*), *π*(*v*) are the covariance matrix, mean vector, and the mixing specification of

 *A*_*i*_(v)  at the tth instant.

#### 3.3.4. Initialization

The GMM is initiated with a Single Cluster.

*C*_1_(1)=(*X*_1_; *δ*_*init*_; 1 : 0) where  *X*_1_*is* the data vector at*t* = 1 and *δ*_*init*_  is the initial covariance matrix whose values are selected from the domain knowledge.

#### 3.3.5. Update

In this subsection, we deduce the equations for updating the GMM *G*(*v* − 1) learned to till the (*v* − 1) *th* to *G*(*v*) with the present data vector  *X*_*V*_. We consider the data vector to be part of the cluster.

*c*_*j*_(*v* − 1)

(6) $$\begin{array}{c} \left(X_{V}-\mu_{j}{\left(v-1\right)}^{T}\delta_{J}{\left(V-1\right)}^{-1}\left(X_{v}-\mu_{j}\left(v-1\right)\right)\right),n\lambda W, \end{array}$$

where *λ* is a user-defined threshold, and *n* is the dimension of the data vector *X* ∈ *R*^*n*^. In the first case, we assume that ∃_*j*_ : *X*_*v*_ ∈ *C*_*j*_(*v* − 1). Let *S*_*i*_(v) be the number of data vectors that have been assigned to  *C*_*i*_(v) till the tth instant. Thus, we have

(7) $$\begin{array}{c} \;\pi_{i}\left(v\right)=\frac{S_{i}\left(v\right)}{v}\\ \pi_{i}\left(v\right)=\frac{\left(v-1\right)\pi_{i}\left(v-1\right)+\delta \left(i-j\right)}{v}\\ \;\pi_{i}\left(v\right)=\left(1-\alpha_{i}\right)\pi_{i}\left(v-1\right)+\alpha_{i}\delta \left(i-j\right), \end{array}$$

where  *α*_*v*_=(1/*v*) and *δ*(*i* − *j*)  is Kronecker's delta.

Now, we update the mean and covariance in *C*_*j*_(*v* − 1) only. To update the mean, we proceed as follows:

(8) $$\begin{array}{c} \;\mu_{i}\left(v\right)=\frac{1}{S_{i}\left(v\right)}\underset{X\in Aj\left(v\right)}{\sum }X\\ \;\mu_{i}\left(v\right)=\frac{s_{j}\left(v-1\right)\mu_{j}\left(v-1\right)+X_{v}}{v\pi_{j}\left(v\right)}\\ \;\mu_{i}\left(v\right)=\left(1\right.-\beta_{j}\left(v\right)\mu_{i}\left(v-1\right)+\beta_{j}\left(v\right)X_{v}. \end{array}$$

where *β*_*j*_(*v*)=*α*_*v*_/*π*_*i*_(*v*).

Similarly, we can update the covariance matrix. From the definition, we can compute the covariance matrix at the t^th^ instant as

(9) $$\begin{array}{c} \;\delta_{j}^{2}\left(v\right)=\frac{1}{S_{j}\left(v\right)}\underset{X\in A_{J\left(V\right)}}{\sum }\left(X-\mu_{j}\left(v\right)\right)\left(X-\mu_{j}\left(v\right)\right){\left(X-\mu_{j}\left(v\right)\right)}^{T}\\ \delta_{j}^{2}\left(v\right)=\frac{1}{S_{j}\left(v\right)}\underset{X\in A_{J\left(V\right)}}{\sum }\left(XX^{T}-\mu_{j}\left(v\right)\mu_{j}{\left(v\right)}^{T}\right). \end{array}$$

Now, further manipulating, by substituting the update rule for *μ*_*j*_(*v*), it can be shown that the updated covariance matrix is given by

(10) $$\begin{array}{c} \delta_{j}^{2}\left(v\right)=\left(1-\beta_{j}\left(v\right)\right)\\ \left(\;\begin{array}{c} \delta_{j}^{2}\left(v-1\right)+\\ \beta_{j}\left(v\right)\left(\left(X_{j}-\mu_{j}\left(v-1\right)\right){\left(X_{i}-\mu_{j}\left(v-1\right)\right)}^{T}\right) \end{array}\right). \end{array}$$

In the second case, it may happen that ∃_*j*_ : *X*_*v*_ ∈ *C*_*j*_(*v* − 1). In such cases, we initialize a new cluster *C*_*k*_(*v*)=(*X*_*v*_; *δ*^2^_*init*_; *α*_*v*_) . If *G*(*v* − 1) has less than *m* clusters, then we add *C*_*K*_(*v*) to it. Otherwise, *C*_*K*_(*v*) changes the cluster with the least weight. In these cases, the mixed specifications of all other clusters are penalized. *π*_*i*_(*v*)=(1 − *α*_*i*_)*π*_*i*_(*v* − 1); *i* ≠ *k*.

### 3.4. Features Selection Using Random Forrest Approach

The Random Forrest (RF) is an integrated learning strategy, which means that it is composed of many tiny submodels, the output of which is combined to form the final output. The RF algorithm is a common machine learning method used for regression, classification, and other learning tasks. The RF algorithm employs a bagging approach to aggregate data from the original dataset. After each group has been trained, the decision tree model is formed. Finally, all of the decision data from the sub-small models are combined and processed to create the final RF model. By utilizing numerous classifiers for voting classification, the RF approach may effectively decrease the error of a single classifier and improve classification accuracy. Practical experience shows that the RF method outperforms artificial neural networks, regression trees, Support Vector Machines, and other algorithms regarding resilience, stability, and classification accuracy. The Random Forrest technique is appropriate for large data processing and may be customized for high-dimensional data. In the lack of data, it may maintain a high classification. The Random Forrest method outperforms other classification algorithms in terms of categorizing efficiency. It can manage massive volumes of data, support massively variable parameters, and easily judge the worth of various features. Many methods and techniques have shown that the Random Forrest approach performs better in classification and is more resilient, consistent, and efficient.

### 3.5. Classification Using CNN Based Upgraded Classifier

In our work, we use CNN, a deep learning-based technique, to examine physical instruction. The best domain in DL applications is CNN, which is made up of pooling, convolutional, and full connection layers. Furthermore, numerous layers, such as the activation function layer, may significantly reduce network training time, enhance networkability, and prevent the dropout layer from overfitting. CNN is a hierarchical model, in which the convolutional layer first retrieves the original data. The dimension reduction data is accepted as the pooling layer's lower convolution input, which then repeats the pooling and convolution process. The source data is supplied based on high-level information. The needed specification is improved by calculating the difference between the absolute and expected values, which is then combined with the backpropagation approach to provide a convergence process. The convolution layer is fundamental to the construction of a convolutional neural network in physical education. After smoothing the input signal using the convolution kernel and filter, it is used to extract local picture properties. Because each convolution kernel's depth matches the input data, the convolution kernel smooths the width and height of the feature map to create a new feature map. The eigenvalues of the first few layers are largely associated with low-order features such as horizontal and vertical edges. In the last levels, low-order qualities are combined to generate high-level aspects. These high-level properties allow these data to be distinguished and mapped to the space for classification. The physical teaching behavior data matrix that has been mapped is

(11) $$\begin{array}{c} \left[\begin{array}{ccccc} M_{11} & M_{12} & . & . & M_{1n}\\ M_{21} & M_{22} & . & . & M_{2n}\\ . & . & . & M_{ij} & .\\ . & . & . & . & .\\ M_{m1} & B_{m2} & . & . & M_{mn} \end{array}\right]. \end{array}$$

The pooling layer's processing specification is constructed using the data matrix obtained from the convolution layer. In contrast to the convolution layer, there is no specification to learn; instead, pick the largest or average value from the targeted region and then construct these highest or mean values into a new feature map. Pooling is a downsampling technique that reduces the number of requirements to reduce network computing complexity. To some degree, it may assist in avoiding overfitting difficulties. Pooling is a technique for reducing the spatial operation of a target region while keeping the same number of input and output data channels. Furthermore, pooling produces the result even if the data changes, improving network stability. At the moment, the outcome of the recognition is as follows:

(12) $$\begin{array}{c} B_{i}^{n+1}=\frac{1}{q}\sum \left[r-q\right]\frac{c}{z}. \end{array}$$

Input the recognized result data to the CNN final layer, the whole connection layer, which integrates all of the preceding layer's picture characteristics and often converts the 2D images formed by convolution into a 1D vector. It is challenging to keep geometric characteristics and then dimensions from highest to lowest while maintaining significant information since the complete connection layer does not retain picture location data. The CNN's complete connection layer uses the feature vector as the classifier's input to acquire the appropriate category's output and identify the original data.

(13) $$\begin{array}{c} D\left(z\right)=\frac{1}{1+e^{v}}. \end{array}$$

The final identification results are denoted by *D* (*z*), while the formula's corrected error value is denoted by *e*. We use a CNN, connection layer, and pooling layer in physical teaching to assess the conduct using the objective function.

### 3.6. Deployment of 5G Network

The teaching method in the 5G network can be constructed using educational theory, merged with an exploration of the usual framework of the education method and the aspects of the 5G network, under the design concepts of teaching physical education. It takes place in a 5G network classroom setting. Students actively seek the need for and understand the essential elements of knowledge and use self-inquiry as the mainstream of educational teaching methods under the guidance of teachers. We effectively utilized the 5G network and incorporated the curriculum under the teacher's supervision, granting students the ability to recognize, analyze, and look online to find design and knowledge through the 5G networks classroom tools.

### 3.7. Data Storing Using Efficient Data Allocation (EDA) Algorithm

When physical teaching resources are stable, the queuing model is utilized to determine the number of copies *m* backlog.

(14) $$\begin{array}{c} \;Q_{SRm=}\lambda_{SRm}R_{SRm=}\overset{N}{\underset{j=1}{\sum }}\lambda_{i}p_{im}\left(R_{\text{wait}}+R_{\text{service}}\right). \end{array}$$

The steady-state copy *m* is obtained based on the utilization ratio of physical teaching, and the number of requests for physical teaching data resources is

(15) $$\begin{array}{c} S_{SRm}=\frac{Q_{SRm}}{\rho_{SRm}}=\frac{\sum_{j=1}^{N}\lambda_{i}P_{im}\left(R_{\text{wait}}+R_{\text{service}}\right)}{\rho_{SRm}}, \end{array}$$

Another optimization goal of the model is to obtain the task of physical teaching resources processing in the entire 5G network platform:

(16) $$\begin{array}{c} s_{\text{total}}\;=\frac{s_{\text{total}}}{\rho_{SRm}\left|S_{SR}\right|}=\overset{M}{\underset{j=1}{\sum }}\overset{\left|S_{SR}\right|}{\underset{m=1}{\sum }}\frac{\lambda_{i}P_{im}T_{SRm}}{\rho_{SRm}}/\left|S_{SR}\right|. \end{array}$$

The physical education resource scheduling problem for 5G networks is abstracted as a multiobjective optimization model in the synthesis: determine the best allocation probability, *p*_im. The average task volume is maximized as a total according to the elasticity of the physical teaching data resource allocation service, and the control function of resource allocation is obtained:

(17) $$\begin{array}{c} \text{Min}R_{\text{total}}=\;\overset{N}{\underset{j=1}{\sum }}\left(\lambda_{i}\right..\frac{\sum_{m=1}^{\left|S_{SR}\right|}P_{im}R_{SRm}}{\sum_{m=1}^{\left|S_{SR}\right|}\lambda_{SRm}}\\ \text{ Max}S_{\text{total}}=\overset{N}{\underset{j=1}{\sum }}\overset{\left|S_{SR}\right|}{\underset{m=1}{\sum }}\frac{\lambda_{i}P_{im}T_{SRm}}{\rho_{SRm}}/\left|S_{SR}\right|\;. \end{array}$$

The optimization technique's main criterion is that the total allocation probability equals 1. Based on the allocation, the allocation of physical teaching resources is maximized.

### 3.8. Glowworm Swarm Optimization

Glowworm Swarm Optimization (GSO) is a technique for concurrently calculating many multimodal function optima. The algorithm outlines the computation that is performed more efficiently by aggregating swarms at optima. Each glowworm in GSO contains its luciferin, which is a bright chemical. A glowworm with a higher luciferin value is better located in the search area and attracts more glowworms. After each iteration, the location of the glowworm will change, as will the luciferin value. The GSO techniques process is as follows:

#### 3.8.1. Luciferin-Update Phase

(18) $$\begin{array}{c} mu_{i}\left(v\right)=\left(1-\varphi \right)m_{i}\left(v-1\right)+\eta Q\left(w_{i\left(v\right)}\right), \end{array}$$

where  *mu*_*i*_(*v*) denotes the updated luciferin value linked with glowworm *i* at time *t*, *φ* is the luciferin decay constant (0 < *φ* < 1), *η* is the luciferin enhanced constant, and *Q*(*w*_*i*(*v*)_) is represented as the objective function of glowworm *i* at time *v*.

#### 3.8.2. Movement Phase

(19) $$\begin{array}{c} Sr_{ij}\left(v\right)=\frac{f_{k}\left(v\right)-f_{k}\left(v\right)}{\sum_{k\in N_{j}\left(v\right)}\left(f_{k}\left(v\right)-f_{i}\left(v\right)\right)}. \end{array}$$

Here, *Sr*_*ij*_(*v*) denotes the probability of movement for a glowworm motion to its neighbor node *j* at time *v*

(20) $$\begin{array}{c} \text{where}j\in N_{i}\left(v\right),\;N_{I}\left(V\right)=\left\{j;d_{ij}\left(v\right)<r_{d}{}^{i}\left(v\right);f_{i}\left(v\right)<f_{j}\left(v\right)\right\}. \end{array}$$

Here, *j* is the set of neighbors of glowworm *i* at the time, *d*_*ij*_(*v*) is the Euclidian distance between glowworm and *k* at time *t*, *r*_*d*_^*i*^(*v*) represents the varying nearby range of glowworm is at time *v* and *f*_*j*_(*v*) is the updated luciferin value.

Then, the discrete-time model of the glowworm movements can be denoted in the following equation:

(21) $$\begin{array}{c} w_{i}\left(v+1\right)=y_{i}\left(v\right)+s\left(\frac{w_{j}\left(v\right)-w_{i}\left(v\right)}{w_{j\left(v\right)}-w_{i\left(v\right)}}\right), \end{array}$$

where *s* is the step-size and estimated as $\;s=\left|d_{ik}-\sqrt{3r}\right|$ and || || denotes the Euclidian norm operator

#### 3.8.3. Neighborhood Range Update Phase

The updated neighborhood range of every glowworm is denoted as

(22) $$\begin{array}{c} r_{d}{}^{i}\left(v+1\right)=\text{min}\left\{r_{s,}\text{max}\left\{0,r_{d}^{i}\left(v\right)+\beta \left(n_{v}-\right.\left|N_{i}\left(v\right)\right|\right\}\right\}. \end{array}$$

where *β* is a constant parameter, and *n* is a parameter used to control the number of neighbors.

In the EEMRGSO algorithm, we used a reverse GSO algorithm for reducing energy consumption. The updated location of sensor *i* is represented *b* the following equation:

(23) $$\begin{array}{c} w_{i}\left(v+1\right)=w_{i}\left(v\right)+\left(G\right.\left(i\;d\right)-\left(w_{i}\left(v\right)\right). \end{array}$$

where  *G*(*i*  *d*)  is the nearest grid-point location from any sensor *i* at time *v*.

#### 3.8.4. Steps of GSO Algorithm

The GSO method takes into account each glowworm's potential solution to the goal issue in space. Glowworms cluster into high-brightness glowworms due to location mobility and mutual attraction, and numerous extreme points in the solution space of a target issue are located. As a consequence, the problem has been rectified. Some of its key points are as follows. (Algorithm 1).

## 4. Performance Analysis

This section elaborates on the results obtained utilizing the suggested approach. Numerous performance metrics may be used to analyze the performance of classification methods based on the accuracy of classification decisions. In a class, variable values can be expected to be either positive (*P*) or negative (*N*) (*N*). The positive cases (*P*) that are properly categorized as positive cases by the methods are referred to as “true positive” (TP) cases, whereas actual positive cases that are incorrectly classified as negative cases by the methods are referred to as “false negative” (FN) cases. Similarly, actual negative cases (*N*) that are correctly labeled as negative cases by the model are considered true negative (TN) cases, whereas actual negative cases that are incorrectly denoted as positive cases by the methods are considered false positive (FP) cases.

### 4.1. Accuracy

It determines how many samples are accurately classified. It determines how closely the outcomes correlate to the original outcome.

(24) $$\begin{array}{c} \text{Accuracy}=\frac{TP+TN}{TP+FP+FN+TN}*100\%. \end{array}$$

Figures 2 and 3 depict a comparison of the accuracy of existing and proposed CNN-based improved classifier techniques. The line graph demonstrates that the suggested technique outperforms the current methods in terms of accuracy.

### 4.2. Precision

It evaluates how precise the suggested method's performance is by analyzing the correct TPs from the anticipated ones.

(25) $$\begin{array}{c} \text{Precision}=\frac{TP}{TP+FP}*100\%\;. \end{array}$$

Figure 4 shows a comparative analysis of the precision for the existing and the proposed CNN-based upgraded classifier methods. The line graph shows that the proposed methodology is more precise than the existing systems.

### 4.3. Recall

The recall is also termed as sensitivity, and it is the fraction of the sum of relevant samples that are obtained.

(26) $$\begin{array}{c} \text{Recall}=\frac{TP}{TP+FN}*100\%. \end{array}$$

Figure 5 shows a comparative sensitivity analysis for the existing and the suggested CNN-based upgraded classifier methods. The line graph shows that the proposed methodology is better than the existing systems.

### 4.4. *F*1 score

*F*1 *score* is a measure of the accuracy of the test. The *F*1 score is calculated by taking the harmonic mean of precision and recall.

(27) $$\begin{array}{c} \;f1\text{ score}=2*\frac{\text{precison}*\text{recall}}{\text{precison}+\text{recall}}. \end{array}$$

Figure 6 shows a comparative analysis of *F*1 score for the existent and the suggested CNN-based upgraded classifier methods. The line graph shows that the proposed methodology is superior to the existing systems.

### 4.5. Throughput

The rate at which data is processed and moved from one location to another is referred to as throughput. It is a term used in networking to describe how well a network performs. Throughput is measured in bits per second or data per second.

Figure 7 shows a comparative analysis of throughput for the existent and the suggested efficient data allocation and Glowworm swarm optimization algorithm. The line graph shows that the proposed methodology is superior to the existing systems.

### 4.6. Memory Utilization

Memory utilization is the fraction of the average amount of memory required to complete a task that is in use at any given time.

Figure 8 portrays a comparative examination of memory utilization for the existent and the suggested efficient data allocation and Glowworm swarm optimization algorithm. The line graph shows that the proposed methodology is superior to the existing systems.

## 5. Conclusion

In this paper, we have suggested a unique method using a CNN-based upgraded classifier for physical education teaching, and the performance metrics such as precision, *f*1 score, accuracy, and recall values are improved compared to the existing approaches. We also utilized a method for optimizing the data allocation for physical teaching resources using the 5G network. The Glowworm swarm optimization proposed is mainly applied to solving data object clustering problems under unsupervised learning conditions. The glowworm swarm optimization is proved to have a better clustering effect and stability. The experimental outcome shows that the memory utilization and throughput are more improved than the existing approaches. [21–27].

## Figures and Tables

**Figure 1:** Schematic representation of the proposed method.

**Figure 2:** Comparison of accuracy (%) for existing and proposed methods.

**Figure 3:** Comparison of accuracy (%) w.r.t accuracy rate.

**Figure 4:** Comparison of precision (%) for the existing and proposed method.

**Figure 5:** Comparison of recall (%) for the existing and proposed method.

**Figure 6:** Comparison of *F*1 score (%) for the existing and proposed method.

**Figure 7:** Comparison of throughput (Mbps) for the existing and proposed method.

**Figure 8:** Comparison of throughput (Mbps) for the existing and proposed method.

**Algorithm 1:** Algorithm for glowworm swarm optimization.

## Data Availability

The data used to support the findings of this study are available from the corresponding author upon request.
